The article "Frederick G Banting (1891-1941): A Pioneer in Diabetes Treatment" was published in 2024. Journal: Cureus.

# Frederick G Banting (1891-1941): A Pioneer in Diabetes Treatment

**DOI:** 10.7759/cureus.73806

**Published:** 2024-11-16

**Authors:** Yash Sharma, Ajith Kannan, James M Lee, Frederick Coffman, Rahul Mittal

**Affiliations:** 1 Health Informatics, Rutgers University, Piscataway, USA; 2 Orthopaedic Surgery, Orange Orthopaedic Associates, West Orange, USA; 3 Biomedical Informatics, Rutgers University, Piscataway, USA

**Keywords:** biographies, historical vignette, historical vignettes, medical innovation, medical stories

## Abstract

The discovery of insulin by Frederick G Banting and his colleagues in 1921 marked a pivotal moment in medical history. Born in Ontario, Canada, in 1891, Banting's childhood was impacted by the death of his closest friend, Jane, who died of diabetes mellitus at a young age. This personal tragedy profoundly influenced him to choose a career in medicine and fueled his determination to find a cure for diabetes. This journey led to the discovery of Insulin with the help of Charles H Best and John JR Macleod, resulting in a Nobel Prize for this work. Their discoveries set the stage for advancements in clinical medicine and biotechnology, including developing recombinant insulin over 50 years later.

## Introduction and background

This review article highlights the work done by Sir Frederick G Banting at the University of Toronto in 1921, which led to the discovery of insulin (Figure 1)[1]. James Collip, a biochemist, also played a crucial role in the discovery by purifying insulin to make it safe for human trials. His contribution was instrumental in discovering insulin, a practical and life-saving treatment for diabetes. The discovery of insulin provided a basic understanding of this endocrine hormone, its function in human physiology, and its role in metabolic regulation, which has led to further research and discoveries in developing slow-acting and potent varieties of insulin. Following Banting's groundbreaking work, he became the youngest person in the world to be awarded the Nobel Prize in Medicine in 1923, which he shared with John James Richard MacLeod. Insulin quickly became the cornerstone of diabetes management.

**Figure 1:** Sir Frederick G. Banting Sir Frederick G. Banting [1], licensed under CC0 1.0

## Review

History serves as the pioneer for all research and development, with evidence of diabetes being traced back over 3,000 years [2]. Diabetes is one of the oldest diseases to have plagued human civilization. However, due to limited anatomical knowledge, an incomplete understanding of bodily processes, and the absence of diagnostic tools, the disease was a profound mystery to early medical practitioners for centuries; nevertheless, physicians didn't miss symptoms like excessive thirst, increased appetite, gradual weight loss, and frequent urine that smelled honey-like, often attracting ants, [3]. These symptoms were recognized, but the underlying cause remained unknown [4]. The discovery of insulin was a turning point in not only understanding diabetes but also dispelling many misconceptions that had clouded the field [5]. Before this, people believed that diabetics needed to eat more, especially sugar, to compensate for the loss of fluids through urination, with some believing herbal remedies and lifestyle, and dietary modifications were enough to cure the condition [6]. The quest for a breakthrough in diabetes treatment persisted, setting the stage for one of the most significant medical discoveries of the 20th century: the isolation and production of insulin. 

Diabetes in history, early observations, and remedies

Before the breakthrough discovery of insulin, historical understandings and treatments of diabetes laid essential groundwork, albeit limited by the knowledge of the time. Ancient Egyptian, Greek, and Indian physicians (Figure 2) had observed symptoms of excessive thirst and frequent urination, attempting various remedies like specific diets to manage symptoms. The earliest records, dating back to around 1552 BCE in Egypt, describe symptoms like excessive thirst and urination in the Ebers Papyrus, one of the oldest medical texts. Ancient Greek physicians, including Hippocrates, observed similar symptoms but could not identify a clear cause, leading to limited and often ineffective treatments [7]. In India and China, diabetes was known as the "honey urine disease," referring to the sweet smell and taste of diabetic urine, and Ayurvedic and Chinese medical texts suggested dietary and herbal remedies to manage it [8].

**Figure 2:** This timeline illustrates the gradual progression in diabetes understanding and treatment, culminating in a pre-insulin era that set the stage for the discovery of insulin and a revolution in diabetes care. The figure is drawn by the authors.

During the medieval period, Islamic scholars advanced the understanding of diabetes further. People like Avicenna, a Persian physician, documented the symptoms of diabetes extensively and advocated for a holistic treatment approach, including diet modification, exercise, and herbal medicine [8]. These medieval Islamic contributions represented a shift towards systematic study and management of diabetes, laying early foundations for the structured approaches that would emerge centuries later [2].

Advancements in understanding diabetes through key discoveries

The 17th and 18th centuries marked important advancements in understanding diabetes, particularly with the discovery of sugar in the urine of diabetic patients. In 1675, English physician Thomas Willis noted the distinct sweetness of diabetic urine, coining the term "diabetes mellitus" to describe this characteristic. This observation shifted the understanding of diabetes from a vague disorder to one involving sugar metabolism. Later, in 1776, British physician Matthew Dobson confirmed the presence of sugar in both the urine and blood of people with diabetes, reinforcing the connection between the disease and elevated blood sugar levels [9]. This marked an important shift, as physicians finally began associating diabetes with sugar metabolism rather than solely viewing it as an imbalance of bodily fluids.

In 1935, French pharmacist Apollinaire Bouchardat made significant contributions to diabetes management by recognizing the link between diet and blood sugar control. Bouchardat observed that diabetes symptoms seemed to improve in patients experiencing food shortages during the Franco-Prussian War (1870-1871) [8]. Based on these observations, he pioneered an early dietary management strategy advocating for strict low-carbohydrate diets to help control symptoms. This relationship between diet and diabetes marked a major step forward and was further evidenced and supported by other practitioners who also advocated for similarly reduced carbohydrate intake and calorie-restricted diets to manage symptoms [9-13]. These approaches laid the groundwork for understanding dietary impacts on diabetes before the advent of insulin therapy.

The 19th century also brought pivotal anatomical discoveries. In 1869, German pathologist Paul Langerhans identified clusters of cells (Figure 3) in the pancreas, later renamed the Islets of Langerhans, which would eventually be linked to insulin production [13]. In 1889, researchers Joseph von Mering and Oskar Minkowski demonstrated that removing the pancreas from dogs induced a significant spike in the dog's blood sugar levels, suggesting a direct role of the pancreas in the disease. These insights provided essential clues about the biological underpinnings of diabetes, setting the stage for the discovery of insulin in the 20th century and transforming diabetes from an often fatal disease into a much more manageable condition [14].

**Figure 3:** Cluster cells (200x magnification, hematoxylin-eosin stain) Islet of Langerhans in human pancreas by phase contrast, licensed under CC0 1.0. Figure is based on research done by the Berkshire Community College Bioscience Image Library [15].

Discovery and impact of insulin

In 1921, Canadian researcher Frederick Banting, building on these previous discoveries, hypothesized that the pancreas was crucial in managing diabetes through its role in protein metabolism. Banting’s work led to the groundbreaking discovery of insulin, which revolutionized diabetes management by enabling patients to effectively regulate their blood sugar levels for the first time [16]. 

Prior to insulin’s introduction in 1922, the prognosis for individuals living with Type 1 diabetes was dire. The literature reports that mortality rates and survival outcomes significantly improved post-insulin [17-19]. Pre-insulin patients generally survived only 1-2 years post-diagnosis despite undergoing dietary treatments and supportive care [17]. For example, data from the Joslin Clinic in Boston show a mortality rate of 824 per 1,000 between 1897-1914, improving to 386 per 1,000 between 1914-1922, right before insulin became available [18].

After insulin's introduction, mortality rates dropped significantly and provided patients with improved survival outcomes [19]. This discovery, however, provided patients with increased chances of survival post-diagnosis [20]. 

Banting’s early life influences 

Frederick Banting’s path to medicine was shaped by two pivotal childhood events. The first was witnessing doctors care for two men injured in a roof collapse, an experience that sparked his desire to help others through medicine. The second was the loss of his childhood best friend, Jane, who developed symptoms of unquenchable thirst and weight loss, now recognized as early signs of diabetes. Jane was an energetic young person who changed after her 14th birthday. She developed an unquenchable thirst and began losing weight, which we now know are the early signs of untreated diabetes. Jane eventually passed away from her illness, and Banting was chosen to be one of her pallbearers [21]. Her death led him to wonder how no doctor had yet found a cure for diabetes fueling his determination to pursue a career in medicine and ultimately inspiring his groundbreaking research into the disease.

Although his family discouraged Banting from entering medicine, he was able to transfer to the University of Toronto Medical School in Toronto, Canada. By 1918, Banting had completed medical school and surgical training and had been awarded a license to practice medicine and surgery by the Royal College of Physicians in London [22]. Due to a downturn in business, Banting worked part-time as a professor at the University of Western Ontario. Since one of his lectures was on the pancreas, he was required to research it thoroughly. This was when he saw an article by Dr. Joseph Freiherr von Mering and Dr. Oscar Minkowski in 1889 that showed that a dog with its pancreas removed showed symptoms similar to those of a diabetic patient. Banting came across a report by Moses Barron titled "The Relation of the Islets of Langerhans to Diabetes," which addressed a critical challenge faced by scientists: isolating the Langerhans islets from the surrounding pancreatic exocrine tissue [22]. This intrigued Banting, which led him to dig deeper, eventually writing down the lines that would change the world and the field of medicine forever. He wrote, "Diabetus [sic]. Ligate pancreatic ducts of dog. Keep dogs alive till acini degenerate, leaving islets. Try to isolate the internal secretion to relieve glycosuria [sic]" [23].

Transitioning from thought to experimentation

After nursing the idea, Banting went to Professor John James Rickard Macleod at the University of Toronto because he needed resources and a lab. However, Banting didn't impress Professor Macleod as Banting did not have a Ph.D. or any research experience. Despite this, he gave Banting a chance, set him up in a small lab, assigned Charles Best as his lab partner, and gave him some experimental dogs. Their initial experiments began in May of 1920 when Banting and Best started testing pancreatic enzyme extracts. One year later, they isolated the islet cells of Langerhans from pancreatic tissue. They did this by tying off the pancreatic duct to shrink the exocrine pancreatic tissue, which usually represents around 95% of the mass of the pancreas. This process allowed them to produce a usable pancreatic extract sample derived primarily from insulin-producing islet cells. They then injected the sample into a dog with its pancreas removed and noted how the dog's blood sugar level dropped (Figure 4) [23].

**Figure 4:** This graph shows the difference in blood sugar levels in Dog 410 after being injected with Insulin and sugar. The blood sugar levels initially dropped after 4cc of insulin extract was injected and increased after sugar was administered through the stomach tube The X-axis shows the time after 4cc of insulin was injected, with approximately two-second intervals. The Y-axis shows the blood sugar levels in mg/dl. The graph was taken from Science Direct. There are no known copyright restrictions on the use of this work [14].

The drop in blood sugar levels led them to believe that the products of the pancreas, more specifically products of the islet cells, had partially isolated and directly correlated with changes in blood sugar levels [23]. After a series of tests, they found correlations between the addition of pancreatic juice and blood sugar levels; however, after they had shown Macleod their work, he was skeptical, mainly because their testing utilized unpurified protein extracts. Macleod's skepticism led to verbal conflicts with Banting, who threatened to take his work elsewhere unless Macleod agreed to an ultimatum: he was allowed to continue his work, got a more extensive lab, and was paid for his experiments. After witnessing the progress of their attempts to isolate Insulin from pooled pancreas tissues taken from larger animals, Macleod taught Banting and Best the methodology of alcohol extraction of proteins, enabling them to produce protein fractions with much higher levels of insulin, which allowed them to give doses with greater potency, and isolate more significant amounts of insulin. With the help of James Collip, Banting and Best were able to purify the insulin extract.

During November and December of 1921, they made significant changes to their approach to insulin purification. They couldn't extract as much insulin as they needed from the dogs, so they began using pancreatic tissues from larger animals obtained from a nearby slaughterhouse. The larger size of these organs, primarily from cows, pigs, and sheep, plus the much larger number of organs that could be obtained, significantly advanced the study of insulin function [24]. Manufacturers in the United States continued to extract insulin from cows until 1982 when the FDA approved the use of cloned insulin [25]. 

Breakthrough in insulin purification and the first human trials

The primary injection in a human patient was given on January 11, 1922, to Leonard Thompson, a 14-year-old Type 1 diabetic. This injection resulted in some reduction in the patient's blood glucose levels. However, the patient's urinary ketone levels were still high, and he developed a sterile abscess at the injection site. Collip worked around the clock, purifying the extract even further, and Leonard was given a second injection on January 23, 1922. This injection was significantly more successful, yielding the following results: Leonard’s blood sugar dropped from 520 mg/dl on January 23 to 120 mg/dl by January 24, ketonuria was eliminated, and glucosuria showed a rapid decrease [26]. This trial was a significant milestone, as it improved his condition and was the basis for the discovery of insulin as the critical element in the disease pathology of Type I diabetes. The success of these trials ultimately paved the way for mass production of insulin. 

Advancements in insulin production

Eli Lilly mass-produced insulin and started shipping them by October 1923 [11]. They initially struggled with increased demands even though the potency varied by up to 25% per lot. So, an isoelectric precipitation method was introduced, leading to a more consistent extraction of more potent insulin, and as a result, the potency varied only about 10% per lot. In 1923, August Krogh, from the University of Copenhagen, talked with Banting and Best since his wife had diabetes, and he wanted to learn more about insulin. He then received permission from the University of Toronto to bring insulin to Scandinavia. Nordisk Insulin Laboratory, a non-profit institution, then started its production [27].

The production of commercial insulin was performed by isolation from animal tissues until the early 1980s when molecular biotechnology had advanced to the point where the cloned gene for human insulin could be expressed in *Escherichia coli* bacteria (by scientists working at Genentech, one of the earliest biotechnology companies). Biologically active forms were successfully isolated from bacterial extracts. The cloning and expression of biologically active insulin, comprising both the A and B chains of the hormone and identical to human insulin in function and immunogenicity, marked a groundbreaking achievement for the biotechnology industry. This innovation fueled the rapid expansion of biotechnology in the 1980s. Genentech partnered with Eli Lilly, a long-time producer of animal-derived insulin, to commercialize this recombinant human insulin (rDNA insulin) and bring it to market. Today, nearly all clinically used insulin is cloned human insulin, and it is estimated that over 2 billion cows would have been required to meet demand if bacterial synthesis had not been developed.

## Conclusions

The discovery of insulin by Frederick Banting, Charles H Best, and JJR Macleod represents one of the most significant medical breakthroughs of the 20th century. The advancement transformed diabetes from a fatal disease into a manageable condition, saving countless lives. Banting's perseverance, innovative thinking, and collaboration with Charles Best, James Collip, and JJR Macleod underscore the importance of interdisciplinary teamwork in scientific discovery. Frederick Banting continued his medical research and held several prominent positions in his lifetime. He became Canada's first professor of medical research at the University of Toronto and directed research at the Banting and Best Department of Medical Research. Banting also explored other areas of interest, including cancer, silicosis, and aviation medicine during World War II. He served as an honorary consulting surgeon at the Toronto General Hospital and the Hospital for Sick Children and remained dedicated to advancing medical science until his death. Banting died in a plane crash on February 21, 1941, at the early age of 49, but the legacy of insulin continues to inspire ongoing research into diabetes treatment and management, reminding us of the profound impact that medical research can have on human health.
